The article "L-Citrulline increases hepatic sensitivity to insulin by reducing the phosphorylation of serine 1101 in insulin receptor substrate-1" was published in 2015. Journal: BMC Complement Altern Med.

# L-Citrulline increases hepatic sensitivity to insulin by reducing the phosphorylation of serine 1101 in insulin receptor substrate-1

**DOI:** 10.1186/s12906-015-0706-4

**Published:** 2015-06-18

**Authors:** Hisae Yoshitomi, Maki Momoo, Xiao Ma, Yewei Huang, Shiori Suguro, Yoshie Yamagishi, Ming Gao

**Affiliations:** School of Pharmaceutical Sciences, Mukogawa Women’s University, 11-68 Koshien Kyuban-cho, 663-8179 Nishinomiya, Hyogo Japan; Key Laboratory of Pu-erh Tea Science, Yunnan Agricultural University, 650201 Kunming, China; College of Life Science, Jilin University, 130012, Changchun, China; Protein Chemical Co., LTD, 1000011 Tokyo, Japan

**Keywords:** Insulin resistance, L-citrulline, Insulin receptor substrate-1, SHRSP.Z-Leprfa/IzmDmcr rat, H4IIE cells

## Abstract

**Background:**

Insulin resistance is characterized by deficient responses to insulin in its target tissues. In the present study, we examined the effects of L-Citrulline (L-Cit) on insulin sensitivity and signaling cascades in rat hepatoma H4IIE cells and SHRSP.Z-Leprfa/IzmDmcr rats.

**Methods:**

H4IIE cells were pretreated in the presence or absence of 250 μM L-Cit in serum-free medium and then incubated in the presence or absence of 0.1 nM insulin. Rats were allocated into 2 groups; a control group (not treated) and L-Cit group (2 g/kg/day, L-Cit) and treated for 8 weeks.

**Results:**

L-Cit enhanced the insulin-induced phosphorylation of Akt in H4IIE cells. Moreover, the inhibited expression of Dex/cAMP-induced PEPCK mRNA by insulin was enhanced by the L-Cit treatment. The phosphorylation of tyrosine, which is upstream of Akt, in insulin receptor substrate-1 (IRS-1) was increased by the L-Cit treatment. The L-Cit-induced enhancement in insulin signaling was not related to the binding affinity of insulin to the insulin receptor or to the expression of the insulin receptor, but to a decrease in the phosphorylation of serine 1101 in IRS-1. These results were also confirmed in animal experiments. In the livers of L-Cit-treated rats, PI3K/Akt signaling was improved by decreases in the phosphorylation of serine 1101.

**Conclusions:**

We herein demonstrated for the first time the beneficial effects of L-Cit on improved insulin resistance associated with enhanced insulin sensitivity. These results may have clinical applications for insulin resistance and the treatment of type-2 diabetes.

## Background

Metabolic syndrome is a lifestyle-related disease caused by a high nutrient condition or lack of exercise. The development of insulin resistance due to obesity has attracted attention as an underlying mechanism for the basic background of metabolic syndrome. Insulin resistance refers to reduced peripheral insulin sensitivity. The binding of insulin to insulin receptors promotes the phosphorylation of insulin receptor substrates (IRS) and activates the intracellular intermediate phosphatidylinositol 3-kinase (PI3K), which, in turn, leads to the phosphorylation of protein kinase B (Akt), a serine/threonine-specific protein kinase [1, 2]. The activation of Akt in the liver inhibits gluconeogenesis by predominantly suppressing the expression of genes for the key gluconeogenic enzymes, phosphoenolpyruvate carboxykinase (PEPCK) and glucose-6-phosphatase (G6Pase). Therefore, insulin resistance in the liver is characterized by deficient responses to insulin, such as enhanced gluconeogenesis [3], which ultimately cause or worsen hyperglycemia. Drug therapy for insulin resistance is a recently developed approach that may improve insulin resistance, but is associated with the risk of side effects, which explains the utility of insulin resistance control by the selection of appropriate foods for safety.

The article "L-Citrulline increases hepatic sensitivity to insulin by reducing the phosphorylation of serine 1101 in insulin receptor substrate-1" was published in 2015. Journal: BMC Complement Altern Med.

L-citrulline (L-Cit) is one of the amino acids that are found in large amounts in cucurbits including the watermelon [4]. Recent studies reported that some amino acid supplementations influence insulin resistance [5, 6]. On the other hand, L-Cit has been shown to play a role in the nitric oxide (NO) system in humans and potentially has antioxidant and vasodilatory effects [7]: however, the effects of L-Cit on insulin resistance have not yet been examined.

We hypothesized that L-Cit may play a role in improving insulin sensitivity via the liver. Therefore, we herein investigated the effects of L-Cit on insulin signaling improvements in rat hepatoma H4IIE cells, which have the ability to produce glucose and have been used to develop an obesity-related insulin-resistant model [8]. We also examined the effects of L-Cit *in vivo* using SHRSP.Z-Leprfa/IzmDmcr rats (SHRSP/ZF), which are resistant to insulin.

## Materials and methods

### Cell culture and treatment

H4IIE cell (DS Pharma Biomedical Co., Ltd.) was used between passage numbers 12 and 45. Cells were cultured in 6-well tissue culture plates (Becton, Dickinson and Company, Japan) and grown to near confluence in Dulbecco's modified Eagle's medium (Nacalai Tesque, Kyoto) containing 10 % fetal bovine serum at 37 °C under a 5 % CO_2_ atmosphere. Cells were pretreated in the presence or absence of 250 μM or 100 μM L-Cit (supplied by Protein Chemical Co., Ltd., Japan) in serum-free medium for 1 h and were then incubated for 10 min in the presence or absence of 0.1 nM insulin. In order to measure phosphoenolpyruvate carboxykinase (PEPCK) gene expression, cells were treated for 6 h with 500nM Dexamethasone and 0.1 mM cAMP (Dex/cAMP) to induce PEPCK gene expression together with 250 μM L-Cit and/or 10 nM insulin during the same time frame.

The article "L-Citrulline increases hepatic sensitivity to insulin by reducing the phosphorylation of serine 1101 in insulin receptor substrate-1" was published in 2015. Journal: BMC Complement Altern Med.

### Binding kinetics assays

We measured the binding kinetics of insulin and INSR using Bio-Layer Inter-Ferometry (BLI) on Octet RED (ForteBio, USA). All interaction analyses were conducted at 30 °C in PBS buffer unless stated otherwise. Sensor tips were pre-wet for 5 min in buffer immediately prior to use, and the microplates used in the Octet were filled with 200 μL of sample or buffer per well and agitated at 1000 g. The experiments comprised 5 steps: 1. Baseline acquisition (120 s); 2. INSR. Loading onto the SA (Streptavidin) sensor (1200 s); 3. Second baseline acquisition (300 s); 4. Association of insulin for the measurement of k_on_ (300 s); and 5. Dissociation of insulin for the measurement of k_off_ (300 s). The concentration of insulin was 2 μM. Baseline and dissociation steps were carried out in buffer with or without 250 μM L-Cit. Association and dissociation responses (nm) were compared with or without 250 μM L-Cit.

### Animals

Five-week-old male SPF (Specific pathogen-free) SHRSP.Z-Leprfa/IzmDmcr (SHRSP-fatty) rats were supplied by Japan SLC (Shizuoka, Japan). All rats were housed in a climate-controlled (temperature; 22 ~ 24 °C, humidity; 40 ~ 60 %) light-regulated room with 12-h light and dark cycles. These rats were fed normal chow (CE-2) for 1 week to stabilize their metabolic condition. SHRSP-fatty rats were allocated into 2 groups; a control group (n = 7, not treated) and L-Cit group (n = 7, administrated 2 g/kg/day L-Cit by free access to water). We referred to a previous study using Amino acid supplemental doses rate from human to animals [28]. We measured water and food intakes as well as the body weights of rats daily.

All rats were sacrificed at the conclusion of the 8-week treatment period after 12 h of fasting. Rats were anesthetized with pentobarbital (65 mg/kg body weight). Blood samples were collected and sera were centrifuged, frozen, and stored at −20 °C until later analyses. Two rats of each group were selected at random and used for formalin perfusion. The tissues were immediately harvested and cleaned to measure tissue weights, and the liver was promptly frozen in liquid nitrogen and stored at −80 °C for western blotting and gene analyses.

All procedures were carried out in accordance with the guiding principles for the care and use of animals in the field of physiological sciences established by the Physiological Society of Japan, and the study was approved by the Ethics Committee of Laboratory Animals at Mukogawa Women’s University.

### Blood analysis

Serum glucose, cholesterol, triglyceride, and free fatty acid levels were measured enzymatically using an assay kit (Wako, Japan). The concentrations of serum aspartate aminotransferase (AST) and alanine aminotransferase (ALT) were measured using the corresponding commercial enzyme kit (Wako, Japan). Serum insulin levels were analyzed using the rat ELISA kit (SHIBAYAGI Co., Ltd. Japan) following the manufacturer’s protocol.

The article "L-Citrulline increases hepatic sensitivity to insulin by reducing the phosphorylation of serine 1101 in insulin receptor substrate-1" was published in 2015. Journal: BMC Complement Altern Med.

### Extraction of membrane protein complexes

Isolated tissues were homogenized in 200 μl TBS (0.025 M Tris–HCl, 0.15 M NaCl, pH7.2) and centrifuged at 1,000 × g for 5 min at 4 °C. Membrane proteins were extracted with the Mem-PER Eukaryotic Membrane Protein Extraction Kit (Thermo, Japan). The viscous phase containing the membrane protein fraction was collected and proteins were purified by precipitation with 10 % trichloroacetic acid. Recovered proteins were mixed with SDS buffer, boiled for 5 min, and loaded onto 12.5 % SDS-PAGE gels.

### Primary and secondary antibodies

Immunoblotting was performed with the following commercially available antibodies: anti-rabbit Akt, anti-rabbit phospho-Akt (Ser473), anti-rabbit IRS-1, anti-rabbit phospho-IRS-1 (Ser307, Ser612, Ser1101), anti-rabbit IgG, and anti-mouse IgG from Cell Signaling Technology (Beverly, MA). Anti-mouse INSRβ, anti-rabbit phospho-IRS-1 (Tyr 989), and anti-goat PI3-kinase p85α were from Santa Cruz Biotechnology. Anti-mouse β-actin was obtained from Sigma (St. Louis, Mo, US).

### Western blot analysis

Cells were homogenized in ice-cold homogenized buffer containing 50 mM Tris–HCl (pH7.4), 100 mM NaCl, 1 % Nonidet-P40, 0.25 % Na deoxycholate, 0.1 % SDS, 1 mM EDTA, 50 mM NaF, 2 mM Na_3_VO_4_, 30 mM Na pyrophosphate, 2 mM PMSF, 1 mM benzamidine, 0.02 g/mL trypsin inhibitor, 0.02 g/mL leupeptin, and 0.02 g/mL aprotinin. After being incubated for 30 min, lysates were centrifuged at 13,000 g for 10 min and supernatants were isolated. The liver tissue was homogenized in ice-cold homogenized buffer. After being incubated for 2 h, lysates were centrifuged at 20,000 g for 20 min and the supernatants were isolated. Proteins were extracted by boiling the tissues in 0.5 mmol/l Tris/HCl, pH6.8, glycerol, 10 % SDS, 0.1 % bromophenol blue, and 2-mercaptethanol. The proteins (25 μg/lean) were electrophoresed using 7.5 %-12.5 % SDS-PAGE gel at 100 V for 2 h. After fractionating, the proteins were transferred onto a PVDF membrane (Amersham Life Science Inc. Buckinghamshire) at 100 mA for 2 h. The membrane was blocked with Blocking One (Nacalai Tesque, Kyoto) for 20 min. After appropriate blocking, the blot was incubated overnight with the primary antibody in antibody solution 1 (Toyobo, Osaka). It was then washed with TTBS and finally incubated for 1 h with a 1:10000 dilution of anti-rabbit, goat, and mouse IgG-horseradish peroxidase. Detection was achieved using an ECL kit (Nacalai Tesque, Kyoto). β-actin was used as an internal control. The densities of the bands were measured using NIH Images.

The article "L-Citrulline increases hepatic sensitivity to insulin by reducing the phosphorylation of serine 1101 in insulin receptor substrate-1" was published in 2015. Journal: BMC Complement Altern Med.

### Real-time PCR

Total RNA was extracted from H4IIE cells and livers using Sepasol-RNA I Super G (Nacalai Tesque, Kyoto). Total RNA from each sample was reverse transcribed to cDNA using the ReverTra Ace qPCR RT kit (Toyobo). The Thunderbird SYBR qPCR Mix was used for the quantitative real-time RT-PCR analysis of the expression of each gene. The primer sequences were as follows: PEPCK sense, 5’-GCA GAG CAT AAG GGC AAG GT-3’, and antisense, 5’-TTG CCG AAG TTG TAG CCA AA-3’; β-actin sense, 5’-GGG AAA TCG TGC GTG ACA TT -3’, and antisense, 5’-GCG GCA GTG GCC ATC TC-3’. Amplification was performed with a real-time PCR system (ABI Prism 7000). Results are expressed as a relative value after normalization to the expression of β-actin.

### Statistical analysis

Data are expressed as the mean ± SEM. Statistical analyses of the data was performed by the Student’s *t*-test between two groups. For multiple comparisons, one-way analysis of variance followed by Tukey's test was determine the significance of differences. A p value of less than 0.05 was considered significant.

## Results

### Effects of L-Cit on insulin signaling in H4IIE cells

We confirmed that 250 μM L-Cit was not cytotoxic using the MTT method (data not shown). Akt is a central enzyme in insulin signaling; therefore, we examined the effects of L-Cit on the phosphorylation of Akt at ser473. The treatment of H4IIE cells with L-Cit did not affect the phosphorylation of Akt in the absence of insulin, but did in the presence of insulin. A pretreatment with L-Cit significantly elevated the phosphorylation of Akt induced by the subsequent 10-min stimulation with insulin (Fig. 1a). PEPCK is an important gluconeogenic enzyme, and its expression is controlled by the insulin-induced phosphorylation of Akt. Moreover, PEPCK gene expression was previously shown to be increased by Dex/cAMP and markedly repressed by insulin in H4IIE cells [9]. H4IIE cells were stimulated with Dex/cAMP in the presence or absence of L-Cit for 6 h. PEPCK gene expression was significantly lower in the L-Cit and insulin treatment groups than in the only insulin group (Fig. 1b). Moreover, the L-Cit treatment enhanced the phosphorylation of Tyr in IRS-1, which is an upstream factor of Akt, in the presence of insulin (Fig. 1c). These results indicated that L-Cit increased insulin sensitivity. We then examined the protein expression of the insulin receptor to determine whether insulin sensitivity increased the effects of L-Cit and if this was related to the expression of the insulin receptor. However, L-Cit did not affect the expression of the insulin receptor in H4IIE cells (Fig. 1d).

The article "L-Citrulline increases hepatic sensitivity to insulin by reducing the phosphorylation of serine 1101 in insulin receptor substrate-1" was published in 2015. Journal: BMC Complement Altern Med.

**Fig. 1:** Effects of L-Cit on insulin signaling in H4IIE cells. H4IIE cells were treated with L-Cit for 1 h and stimulated for 10mins with 0.1nM insulin. **a** Phosphorylation level of Akt at serine 473, (**b**) PEPCK mRNA level, (**c**) phosphorylation level of IRS1 at tyrosine, (**d**) protein level of IR. Data were expressed as the mean ± SEM of three independent experiments. Significant differences were identified by Tukey’s test, #*p* < 0.05 vs control, *p < 0.05 vs with insulin

### Effects of L-Cit on insulin and its receptor binding

Affinities (K_D_) were calculated from a non-liner global fit of the data between the insulin receptor and insulin in the presence or absence of L-Cit using the Octet software. The KD (M) of the insulin receptor and insulin was 5.72E-07. The KD (M) of the insulin receptor and insulin with L-Cit was 4.78E-07. L-Cit had no significant effect on the insulin binding affinities of the insulin receptor (Fig. 2).

**Fig. 2:** Effects of L-Cit on insulin and its receptor binding. Affinities (K_D_) were calculated from a non-liner global fit of the data between the insulin receptor and insulin in the presence or absence of L-Cit using the Octet software

### Effects of L-Cit on the phosphorylation of serine in IRS-1 in H4IIE cells

IRS-1 plays an important role in insulin signaling. The phosphorylation of Ser in IRS-1 reduces its ability to associate with the insulin receptor, leading to a reduction in insulin signaling. In the present study, no significant difference was observed in IRS-1 ser307 (Fig. 3a) or 612 (Fig. 3b) in the presence or absence of L-Cit. However, the phosphorylation of IRS1 ser1101 was weaker in L-Cit-treated H4IIE cells than in non-treated cells in the presence of insulin (Fig. 3c), whereas no significant difference was observed in the absence of insulin.

**Fig. 3:** Effects of L-Cit on the phosphorylation of serine in IRS-1 in H4IIE cells. H4IIE cells were treated with L-Cit for 1 h and stimulated for 10mins with 0.1nM insulin. **a** Phosphorylation level of IRS1 at serine 307, (**b**) IRS1 at serine 612, (**c**) IRS1 at serine 1101. Data were expressed as the mean ± SEM of three independent experiments. Significant differences were identified by Tukey’s test, #*p* < 0.05 vs control, *p < 0.05 vs with insulin

### Effects of L-Cit supplementation on insulin signaling in SHRSP/ZF rat livers

The results obtained in SHRSP/ZF rats were consistent with those in H4IIE cells. No significant differences were observed in the phosphorylation of IRS-1 Ser307 and 612 in the liver between the groups (Fig. 4a, b). However, the phosphorylation of Ser1101 in IRS-1 was markedly decreased in the L-Cit group (Fig. 4c). PI3K is a downstream factor of IRS-1 and controls the phosphorylation of Akt. PI3K exhibits its effects by translocating to the cell membrane from the cytoplasm [10, 11]. The ratio of cell membrane PI3K was significantly higher in the L-Cit group than in the control group (Fig. 4d). Furthermore, the level of phosphorylation of Akt in the liver was significantly higher in the L-Cit group than in the control group (Fig. 4e). PEPCK gene expression was slightly decreased in the L-Cit group (Fig. 4f). No significant difference was observed in the protein expression of the insulin receptor between the two groups.

The article "L-Citrulline increases hepatic sensitivity to insulin by reducing the phosphorylation of serine 1101 in insulin receptor substrate-1" was published in 2015. Journal: BMC Complement Altern Med.

**Fig. 4:** Effects of L-Cit supplementation on insulin signaling in SHRSP/ZF rat livers. Six-week-old male SHRSP/ZF rats were administrated 2 g/kg/day L-Cit for 8 weeks. At the end of the administration period, the livers were immediately harvested for western blotting. **a** Phosphorylation level of IRS1 at serine 307, (**b**) IRS1 at serine 612, (**c**) IRS1 at serine 1101, (**d**) membrane PI3K level, (**e**) phosphorylation level of Akt at serine 473, (**f**) PEPCK mRNA level. Data were expressed as the mean ± SEM of n = 5. Significant differences were identified by the *t*-test, *p < 0.05, **p < 0.01 vs control group

### Animal characteristics

Table 1 shows that supplementation with L-Cit did not affect food intake or body weight. However, fasting glucose levels were approximately 23 % lower in the L-Cit group than in the control group 8 weeks after the administration of L-Cit, whereas serum insulin concentrations were similar in the two groups. No significant differences were observed in triglyceride, cholesterol, or FFA levels between the groups. AST and ALT also did not differ significantly among the groups during the experimental period.

**Table 1:** Effects of L-Citrulline on metabolic parameters in SHRSP/ZF rat

		Control (n = 7)	L-Citrulline (n = 7)
food intake (g)	0w	24.0 ± 0.5	24.7 ± 0.4
	4w	29.9 ± 0.5	29.4 ± 0.3
	8w	30.5 ± 2.2	29.5 ± 2.6
2.6body weight (g)	0w	121.9 ± 5.9	127.3 ± 4.2
	4w	330.7 ± 4.4	339.4 ± 7.6
	8w	420.5 ± 5.9	415.0 ± 12.2
serum			
insulin (ng/mL)		8.1 ± 3.6	10.8 ± 2.7
glucose (mg/dL)		280.2 ± 35.3	213.9 ± 16.6
triglyceride (mg/dL)		598.7 ± 99.5	594.4 ± 66.1
cholesterol (mg/dL)		94.6 ± 3.5	101.7 ± 3.0
free fatty acid (mEq/L)		1.8 ± 0.4	2.1 ± 0.4

## Discussion

The main result of the present study was that L-Cit increased insulin sensitivity in rat hepatoma H4IIE cells and SHRSP/ZF rats. The underlying mechanism was identified as the stimulation of insulin signaling due to the inhibited phosphorylation of serine1101 in IRS1.

The article "L-Citrulline increases hepatic sensitivity to insulin by reducing the phosphorylation of serine 1101 in insulin receptor substrate-1" was published in 2015. Journal: BMC Complement Altern Med.

Insulin is secreted by the pancreas in response to eating or other stimuli and functions to control blood glucose levels. The binding of insulin to insulin receptors leads to the phosphorylation of tyrosine in IRS, which activates PI3K and subsequently phosphorylates Akt [12]. Akt is an important factor in insulin signaling and the control of glucose metabolism. Phosphoenolpyruvate carboxykinase (PEPCK) is a rate-limiting enzyme that catalyzes hepatic gluconeogenesis. Insulin has been shown to suppress the transcription of PEPCK by activating Akt [13]. In the present study, we demonstrated that L-Cit enhanced the insulin-induced phosphorylation of Akt and reduced PEPCK mRNA expression. We also showed that L-Cit increased the phosphorylation of tyrosine in IRS1, which is upstream of Akt, and this was not related to the binding affinity of insulin to its receptor or the expression of the insulin receptor.

In contrast to the phosphorylation of tyrosine, IRS1 is known to be phosphorylated at many serine sites. Recent studies reported that serine phosphorylation played an important role as a mechanism that negatively regulated insulin signaling [14, 15]. The phosphorylation of serine in IRS-1 may suppress insulin signaling by downregulating the expression of the IRS1 protein through ubiquitination [16], thereby inhibiting the interaction between the insulin receptor and IRS1 phosphotyrosine binding domain [17, 18]. Many stimulators of IRS-1 serine phosphorylation have been identified to date, for example, TNFα and FFA. TNFα phosphorylates serine 307, 612, and 636 in IRS-1 through the activation of several serine kinases including inhibitory-kappa-B kinase [19], JNK [20], and mTOR [21]. FFA activates IKK or JNK and phosphorylates IRS-1 serine 307. On the other hand, FFA stimulates phosphorylation of serine 1101 through PKCθ. A previous study reported that an insulin stimulation also phosphorylated not only IRS1 on tyrosine sites, but also that on serine residues such as Ser307, Ser612, and Ser1101 [22]. This is part of the negative-feedback mechanism induced by insulin. Therefore, insulin resistance may be induced by high insulin level. In the present study, we showed that the insulin stimulation increased the phosphorylation of Ser307 and 612. We observed that the phosphorylation of Ser1101 was increased by the stimulation of insulin, but, devoid of statistical significance. This may be due to high expression of IRS-1 serine1101 phosphorylate form on H4IIE cell in normal condition. However, the activation of general IRS1 may be controlled more by negative feedback. Our results showed that the phosphorylation of Ser1101 was weaker in L-Cit-treated H4IIE cells than in non-treated cells and its effects were detected in the presence of insulin. No significant differences were observed in IRS-1 ser307 and 612 in the presence or absence of L-Cit. These results indicated that L-Cit diminished the inactivation of IRS1 from insulin negative-feedback by decreasing phosphor-IRS-1 ser1101.

The article "L-Citrulline increases hepatic sensitivity to insulin by reducing the phosphorylation of serine 1101 in insulin receptor substrate-1" was published in 2015. Journal: BMC Complement Altern Med.

Thus, we conducted an additional experiment using rats to confirm the insulin resistance-improving effects of L-Cit *in vitro*. SHRSP/ZF which was generated as a new model of metabolic syndrome by crossing SHRSP rats with Zucker Fatty rats. SHRSP/ZF rats become obese, hyperlipidemic, and resistant to insulin due to a mutated leptin receptor [23]. Hence, these rats were characteristically associated with hyperinsulinemia. When insulin levels remain elevated for a long period of time, the phosphorylation of serine in IRS1 may trigger insulin resistance in cells. The phosphorylation of serine residues in IRS1 was previously reported to be increased in models of insulin resistance and type-2 diabetes [24]. The results of the present study were consistent with *in vitro* findings in which PI3K/Akt/PEPCK signaling in the liver was improved by the L-Cit treatment. Furthermore, only the phosphorylation of Ser1101 in IRS-1 was decreased.

Various studies have shown that there is considerable crosstalk between insulin signaling and amino acids. For example, early studies reported that the plasma concentrations of branched-chain amino acids were elevated in obese insulin-resistant subjects [25]. In contrast, Tremblay indicated that amino acid-induced insulin resistance was linked to the S6K1-mediated phosphorylation of Ser1101 in IRS-1 [26]. Ser1101, the unphosphorylated form of IRS-1, enhanced the insulin-induced tyrosine phosphorylation of IRS-1 and Akt Ser473 phosphorylation. We also found that L-Cit supplementation decreased the phosphorylation of Ser1101 in IRS1; however, the molecular mechanisms responsible for this decrease currently remain unclear.

In summary, we herein demonstrated for the first time the beneficial effects of L-Cit on improved insulin resistance associated with enhanced insulin sensitivity through the activation of IRS1 followed by the inhibition of serine 1101 phosphorylation both *in vivo* and *in vitro* (Fig. 5). L-Cit is a naturally occurring amino acid and widely may exist for different tissue. Few studies have demonstrated on the toxicology of supplemental L-Cit, it is generally recognized as safe for oral administration [27]. These results may have clinical applications for insulin resistance and the treatment of type-2 diabetes without side effects.

The article "L-Citrulline increases hepatic sensitivity to insulin by reducing the phosphorylation of serine 1101 in insulin receptor substrate-1" was published in 2015. Journal: BMC Complement Altern Med.

**Fig. 5:** Schematic overview showing the beneficial effects of L-Cit on improved insulin resistance associated with enhanced insulin sensitivity through the activation of IRS1 followed by the inhibition of serine 1101 phosphorylation. Arrows indicate positive inputs (activation), whereas perpendicular lines show negative inputs (inhibition)

## Abbreviations

Akt: Protein kinase B
ALT: Alanine aminotransferase
AST: Aminotransferase
Dex: Dexamethasone
FFA: Free fatty acid
G6Pase: Glucose-6-phosphatase
IKK: IκB kinase
IRS: Insulin receptor substrates
JNK: c-Jun N-terminal kinase
L-Cit: L-Citrulline
mTOR: Mammalian target of rapamycin
PI3K: Phosphatidylinositol, 3-kinase
PKC: Protein kinase C
S6K1: S6 kinase 1
SHRSP/ZF: SHRSP.Z-Leprfa/IzmDmcr
TNFα: Tumor necrosis factor alpha
